# Study on the Relationship between AAD and Clinical Features in Emergency Ward Patients and the Application Effect of Probiotics

This article has been retracted.

**DOI:** 10.1155/2022/6164843

**Published:** 2022-07-11

**Authors:** Wenjuan Qiu, Fangfang Bai

**Affiliations:** Emergency Department, Zhejiang Hospital, Hangzhou 310030, China

## Abstract

In order to investigate the influencing factors of AAD in the emergency ward and the clinical effect of probiotics, 100 AAD patients admitted to the emergency ward of our hospital from January 2021 to January 2022 and 100 healthy physical examination subjects are selected for conducting clinical trials. The subjects are, respectively, included in the AAD group and the healthy group. By using the random number table method, 100 patients in the AAD group are randomly divided into the probiotic group and traditional group, with 50 patients in each group. The traditional group receives conventional treatment, and the probiotic group is treated with *Clostridium* caseinate bifidobacterial probiotics additionally. Multivariate logistic analysis is performed on the risk factors for AAD, and the comparison of tumor necrosis factor-*α* (TNF-*α*), interleukin-6 (IL-6), and the intestinal microflora of the different groups before and after treatment is conducted. The experimental result reveals that probiotics treatment for AAD patients can reduce inflammatory response and promote intestinal colonization of beneficial bacteria such as bifidobacteria.

## 1. Introduction

Antibiotics are chemical substances used by microorganisms to resist the invasion of other microorganisms in the environment and protect their own safety. Antibiotics can kill and inhibit the pathogenic bacteria invading the human body and then control infection and recover the body. Generally speaking, antibiotics are effective against various bacteria, such as chlamydia, mycoplasma, *Rickettsia*, spirochetes, and some human parasitic protozoa, but not against viruses, fungi, and most parasitic infections. The main mechanisms of action of antibacterial drugs are interfering with the synthesis of bacterial cell wall, destroying bacterial cell membrane, blocking bacterial protein synthesis, affecting nucleic acid metabolism, and inhibiting bacterial folate metabolism. Therefore, the use of antibiotics is very common. However, it should be noted that the use of antibiotics will lead to intestinal diseases, resulting in diarrhea, sepsis, and other complications [1].

The occurrence of antibiotic-associated diarrhea (AAD) is closely related to the use of antibiotics, and the incidence rate is increasing year by year. Diarrhea is the main clinical symptom of AAD. The etiology and pathogenesis of antibiotic-associated diarrhea is complex and not yet fully understood. Most researchers believe that the use of antibiotics destroys the normal intestinal flora, and it is the main cause of diarrhea. Some patients may have nausea, vomiting, abdominal pain, and fatigue. Severe patients will have multiple organ failure, which seriously threatens the patient's life, health, and quality of life [2]. Intestinal flora imbalance and inflammatory reaction are related to the occurrence of AAD. Regulating the host intestinal flora is a good clinical treatment for AAD [3]. In recent years, probiotics have been gradually applied to clinical diarrhea and infectious diseases. Among them, *Clostridium* caseinate bifidobacterium powder is widely used. The clinical anti-inflammatory effect of this drug has been recognized. It can improve intestinal flora disorder through various mechanisms [4, 5].

At present, there are few literature studies on the treatment of AAD with *Clostridium butyricum* double active powder. Therefore, the purpose of this study is to analyze the risk factors of AAD in emergency ward patients and the therapeutic effect of probiotic *Clostridium butyricum* double active powder, so as to provide a new idea for the follow-up clinical treatment optimization of AAD.

This paper is organized as follows.  Section 2 discusses the related work, followed by the data and methods in Section 3. In section 4, the results and analysis are proposed. Finally, in Section 5, some concluding remarks are made.

## 2. Related Work

The clinicopathological mechanism of AAD has not been determined yet. The view that the use of antibiotics destroys the balance of intestinal flora and causes AAD has been accepted by most medical researchers [6]. *Clostridium difficile* is the main bacterium that induces AAD, accounting for about 25%. Therefore, the application of probiotics and other effective treatment schemes to intervene and regulate the balance of intestinal flora expression and inflammatory response in AAD patients has certain research value [7].

Ma et al. [8] showed that the increase in age of elderly patients is a risk factor for the occurrence of AAD. The reason is that the increase in age of patients leads to immune function, physiological function, metabolic disorders, and gastrointestinal disorders. For example, the intestinal symbiosis of patients is damaged after antibiotic treatment. To some extent, AAD patients in emergency wards are selected as the research objects. Although AAD can occur at any time point from clinical treatment to 2 months of antibiotic exposure, children have lower gastric acid than adults. In addition, the underdeveloped immune system makes the level of immunoglobulin (Ig) and complement unable to reach the normal level, which leads to intolerance to external environmental stimuli and antibiotics, and indirectly increases the risk of AAD during the effective period of antibiotic exposure. Therefore, children are at high risk of AAD. The above research takes the elderly patients as the research object and analyzes the influencing factors of AAD. However, the therapeutic effect of probiotics needs to be further improved. The physical conditions and states of the elderly and children are different. The related influencing factors and molecular mechanisms of AAD in children in emergency ward need to be further analyzed [9].

Ma et al. [10] demonstrated that the combined use of antibiotics and long-term use of antibiotics would increase the risk of AAD, which was consistent with the results of this study. According to the results of multivariate regression analysis of this study, the combined use of more than two antibiotics and the duration of antibiotic use ≥7 days were independent risk factors for AAD. This indicates that the overuse of antibiotics will increase the clinical risk of AAD. The main reason for this result is that both the combined use of antibiotics and the long-term use of antibiotics can cause intestinal microbiome disorder and abnormal changes in intestinal nutrient metabolism, destroy the normal distribution of intestinal flora, inhibit the proliferation of probiotics in the intestinal flora, and promote the proliferation of pathogenic bacteria, thus leading to intestinal microbiome disorder. In addition, the digestion and absorption of the intestinal tract will affect and destroy the intestinal mucosal barrier and cause diarrhea. Excessive use of antibiotics will produce toxic effects or cause allergies, which will increase the atrophy of intestinal epithelial cilia and damage the intestinal mucosa. In an indirect way, it can inhibit the enzyme activity in the cells and eventually cause the absorption barrier diarrhea [11]. It is suggested that, in the subsequent clinical application of antibiotics in patients, the dosage of antibiotics should be strictly controlled, antibiotic treatment plan should be rationally formulated, and the combined application of multiple antibiotics or long-term application should be avoided as far as possible, so as to reduce the risk of AAD. The results of this study showed that the application of probiotics was a protective factor for the occurrence of AAD in patients, which was consistent with the results of previous research literature [12]. Analysis of the reason may be probiotics can promote intestinal peristalsis which, in turn, stimulates patients' specific immune and nonspecific immune mechanism and thus enhance the intestinal mucosal immunity and the body engraftment resistance, effectively improve the intestinal flora disturbance, further strengthen intestinal barrier, and reduce the risk of pathogen invasion induced AAD.

TNF-*α* is a typical cytokine that can promote inflammatory response. TNF-*α*can promote the secretion of inflammatory factor IL-6 and trigger an inflammatory cascade, which further aggravates intestinal mucosal injury and secretes a large number of inflammatory mediators, ultimately leading to diarrhea [13]. Giuliano et al. [14] showed that the application of probiotics in AAD treatment can stimulate the immune response of the body, thus inhibiting the inflammatory response and improving intestinal diseases by enhancing immunity. Probiotics can be the expression of inflammatory cytokines, which inhibit intestinal epithelial cell apoptosis. At the same time, it can promote the expression and secretion of recombinant mucin 2(MUC2), so as to reduce the damage of intestinal mucosal barrier caused by antibiotics and improve the clinical symptoms of patients [15]. The use of probiotics can promote the implantation of beneficial bacteria such as bifidobacteria and lactobacilli and promote the distribution of the composition and structure of the intestinal flora. In addition, the correct use of antibiotics can avoid intestinal disorders, enhance the diversity and stability of the intestinal flora, and reduce the clinical risk of intestinal diseases caused by AAD [16].

## 3. Data and Methods

### 3.1. General Information

A total of 100 AAD patients admitted to the emergency ward of our hospital from January 2021 to January 2022 were selected as the research object, and 100 healthy people who underwent physical examination during the same period were selected as the control and were included in the case group and the healthy group. The AAD group was randomly divided into the probiotic group and traditional group according to the number table method, with 50 patients in each group. The probiotic group was 56–67 years old, with an average age of 62.11 ± 2.21 years. Body mass index (BMI) was 18–27 kg/m^2^, with an average age of (23.21 ± 2.79) kg/m^2^. There were 10 cases of hypertension, 7 cases of coronary heart disease, and 3 cases of diabetes. The traditional group was 56 to 67 years old, with a mean of 62.11 ± 2.19 years old. BMI was 18 to 26 kg/m^2^, with a mean of 22.89 ± 2.91 kg/m^2^. There were 11 cases of hypertension, 9 cases of coronary heart disease, and 3 cases of diabetes. There were no statistically significant differences in gender, age, BMI, underlying diseases, and other baseline data between the two groups (*P* > 0.05), indicating comparability.

Inclusion criteria are as follows:

1. In line with the diagnostic criteria of AAD
2. Have a history of antibiotic treatment and diarrhea after antibiotic administration
3. Daily stool time is ≥5 times
4. Complete clinical data

Exclusion criteria are as follows:

1. Diarrhea caused by bacterial dysentery, acute attack of chronic enteritis, or food poisoning
2. Intestinal dysfunction
3. The presence of immune dysfunction or immune systemic diseases
4. Incomplete clinical data affecting the accuracy of research data

The purpose, significance, and process of the study have been explained in detail to the patients participating in the study. Informed consent has been signed on the basis of patient resources. The study has been reviewed and approved by the Medical Ethics Committee of the hospital.

### 3.2. Proposed Methods

#### 3.2.1. Treatment Methods

Both groups were given basic treatment such as montmorillonite powder and electrolyte correction, and 1 bag of montmorillonite powder was taken 3 times a day (Baf-Ipsen (Tianjin) Pharmaceutical Co., Ltd., National Drug Approval word H20000690). Patients in the probiotic group were given 1 bag of *Clostridium* caseinate bifidobacterium powder (Shandong Sinovac Biological Products Co., Ltd., National Drug Approval word S20020014) every day, divided 2 times.

#### 3.2.2. Detection Methods of Inflammatory Factors

Before treatment and after fasting for 12h on 7d and 14d, 5 ml of fasting venous blood in the morning was collected by sterile vacuum coagulation tube. After standing for 20 min, centrifugation was carried out for 15 min according to set parameters such as centrifugal force 1000 × g, radius 11 cm, and rotational speed 3000 r/min. Supernatant was divided into centrifugal tubes. Store in refrigerator at −80°C for later use. Tumor necrosis factor alpha (TNF-*α*) and interleukin-6 (IL-6) were detected by enzyme-linked immunosorbent assay (ELISA).

#### 3.2.3. Intestinal Bacteria Detection Method

Stool samples were collected from the patients before treatment and at 7d and 14d of treatment. 1 mL of stool samples was taken and added to 9 mL of sterilized normal saline, fully shaken and inoculated in MRS medium, and incubated at 35–37°C for 72 h. The number of intestinal bifidobacteria and lactobacilli was counted by colony morphology. MRS Petri dish inoculation was carried out in strict accordance with the instructions.

### 3.3. Observation Indicators

The observation indicators include the following:

1. A self-designed clinical information questionnaire was used to analyze the basic information of the subjects, including age, gender, underlying diseases, proton pump inhibitors, fasting, types of antibiotic use, duration of antibiotic use, probiotics, and univariate analysis of baseline data differences between the AAD group and the healthy group
2. Multivariate logistic regression analysis of the influencing factors of AAD in emergency ward patients
3. The levels of TNF-*α*and IL-6 before treatment and 7d and 14d after treatment were detected and compared
4. The number of *Bifidobacterium* and *Lactobacillus* before treatment and 7d and 14d after treatment was detected and compared

### 3.4. Statistical Methods

SPSS 24.0 software was used for statistical analysis. The measurement data of normal distribution were expressed by (*‾x* ± *s*) and *t*-test. Multiple groups of data were tested by *F* test. Mauchly test was used for comparison of data at different time points within the group. *P* > 0.05 indicated that the covariance matrix was full of football symmetry, and the percentage of counting data *n* (%) indicated that the *X*^*2*^ test was used. Multivariate logistic regression analysis of the influencing factors of AAD in emergency ward patients is conducted, and the difference was statistically significant.

## 4. Experimental Results and Analysis

### 4.1. Univariate Analysis of Clinical Data Differences between the AAD Group and the Healthy Group

There were no statistically significant differences in gender, combined underlying diseases, proton pump inhibitors, fasting, and other clinical data between the two groups (all *P* > 0.05). The incidence of AAD in AAD group was significantly higher than that in healthy group with age ≥65 years, antibiotic use ≥2 kinds, and antibiotic use time ≥7d. The incidence of AAD in the AAD group using probiotics was significantly lower than that in the healthy group with statistical significance (*P* < 0.05), as shown in Table 1.

### 4.2. Multivariate Logistic Regression Analysis of Risk Factors for AAD

Factors with *P* < 0.05 and the occurrence of AAD in the emergency ward were taken as independent and dependent variables respectively, and variable assignment values are shown in Table 2. Multivariate logistic regression analysis showed that age ≥65 years, antibiotic use ≥2 types, and antibiotic use duration ≥7d were independent risk factors for AAD in emergency ward patients. Besides, the probiotics were protective factors, as shown in Table 3.

### 4.3. Comparison of TNF-*α* and IL-6 Levels before and after Treatment

The levels of TNF-*α* and IL-6 in both groups showed a decreasing trend after treatment, and the levels of TNF-*α* and IL-6 in probiotics group were lower than those in the traditional group after 7d and 14d. The differences were statistically significant (*P* < 0.05), as shown in Table 4 and Figure 1. A, B, and C represent the comparison with other time points, respectively. In addition, the symbol “#” represents the comparison with the traditional group (*P* < 0.05).

### 4.4. Comparison of Intestinal Flora Changes before and after Treatment

The number of *Bifidobacterium* and *Lactobacillus* in the two groups showed an increasing trend after treatment, and the number of *Bifidobacterium* and *Lactobacillus* in the probiotic group was higher than that in the traditional group 7d and 14d after treatment. The differences were statistically significant (*P* < 0.05), as shown in Table 5 and Figure 2.

## 5. Conclusions

In this study, the influencing factors of AAD in emergency ward and the clinical effect of probiotics is investigated. From the results, it can be observed that the age, probiotics, antibiotic combination, and duration of antibiotic use will affect the incidence of AAD in emergency ward patients. The individualized and rational antibiotic treatment should be formulated for patients. In addition, probiotics can significantly improve the inflammatory response and promote the colonization of intestinal beneficial flora in patients with AAD, which is helpful to correct intestinal disorders in patients with AAD. Also, our study still has certain limitations in aspects of small sample size and incomplete inclusion of factors in clinical single-factor analysis. In the future, we should expand the sample size and refer to the literature to include other clinical factors related to the occurrence of AAD for indepth study with large sample size and multicenter.

## Figures and Tables

**Figure 1:** Levels of inflammatory factors at different time points: (a) TNF-*α*; (b) IL-6.

**Figure 2:** Changes of intestinal flora at different time points: (a) *Bacillus bifidus*; (b) *Bacillus lactis*.

**Table 1:** Univariate analysis of clinical data differences between the AAD group and the healthy group (*n*, %).

Factor	AAD group (*n* = 100)	Healthy group (*n* = 100)	*X* ^*2*^	*P* value
Sex				

Male	44	48	0.322	0.570
Female	56	52		

Age (years)				

<65	32	46	4.119	0.042
≥65	68	54		

Combined with basic diseases				

Yes	43	47	0.323	0.570
No	57	53		

Jejunitis				

Yes	52	49	0.180	0.671
No	48	51		

Proton pump inhibitor				

Yes	47	44	0.181	0.670
No	53	56		

Types of antibiotic use (species)				

<2	27	65	29.066	<0.001
≥2	73	35		

Time of antibiotics use (d)				

<7	31	45	4.160	0.041
≥7	69	55		

Probiotics				

Yes	35	78	37.616	<0.001
No	65	22		

**Table 2:** Variable assignment.

Factor	Variable name	Assignment
Types of antibiotic use (species)	*X1*	≤2 = 1, >2 = 2
Age (years)	*X2*	<65 = 1, ≥65 = 2
Time of antibiotics use (d)	*X3*	<7 = 1, ≥7 = 2
Probiotics	*X4*	Yes = 1, No = 2
AAD occurred in the emergency ward	*Y*	No = 1, Yes = 2

**Table 3:** Multivariate logistic regression analysis of influencing factors of AAD in emergency ward patients.

Influencing factor	*B* value	SE value	Wald value	*P* value	OR value	95%CI
There were >2 types of antibiotics used	1.117	1.407	0.631	0.030	3.078	1.195∼8.782
Age ≥65 years	3.429	1.293	7.041	0.007	3.835	2.449∼11.015
Time of antibiotic use ≥7d	2.947	1.306	5.100	0.022	3.063	1.468∼16.443
Probiotics	−4.254	2.323	3.557	0.025	1.256	0.951∼9.246

**Table 4:** Comparison of TNF-*α*and IL-6 changes before and after treatment (‾*x* ± s).

Group	Time point	TNF-*α* (ng/L)	IL-6 (ng/L)
Probiotic group (*n* = 50)	Pretherapy	18.20 ± 2.41	55.29 ± 7.82
	After 7d of treatment	14.22 ± 2.34	31.11 ± 5.42
	After 14d of treatment	9.21 ± 1.13	21.21 ± 3.16

Traditional group (*n* = 50)	Pretherapy	18.17 ± 2.39	55.31 ± 7.79
	After 7d of treatment	16.29 ± 2.31	42.41 ± 6.45
	After 14d of treatment	11.41 ± 1.20	35.71 ± 4.22

*F*_time point_		3545.754	1372.614

*P*_time point_		<0.001	<0.001

*F*_point_ *∗*_group_		765.446	828.412

*P*_point_ *∗*_group_		<0.001	<0.001

**Table 5:** Comparison of changes of the intestinal flora before and after treatment (‾*x* ± s).

Group	Time point	*Bacillus bifidus* (Ig CF/g)	*Bacillus lactis* (Ig CF/g)
Probiotic group (*n* = 50)	Pretherapy	8.31 ± 0.32	9.21 ± 0.62
Traditional group (*n* = 50)	After 7d of treatment	10.11 ± 0.41	11.01 ± 0.72
	After 14d of treatment	11.21 ± 0.46	12.21 ± 0.76
	Pretherapy	8.31 ± 0.32	9.18 ± 0.59
	After 7d of treatment	9.31 ± 0.39	10.28 ± 0.75
	After 14d of treatment	10.71 ± 0.43	11.31 ± 0.72
*F*_time point_		3533.645	1345.609
*P*_time point_		<0.001	<0.001
*F*_point_ *∗*_group_		756.321	825.412
*P*_point_ *∗*_group_		<0.001	<0.001

## Data Availability

The simulation experiment data used to support the findings of this study are available from the corresponding author upon request.

## References

[1] Shi X., Li H. (2013). Anticoagulation therapy in patients with chronic obstructive pulmonary disease in the acute exacerbation stage. *Experimental and Therapeutic Medicine*.

[2] Dinleyici M., Vandenplas Y. (2019). *Clostridium difficile* colitis prevention and treatment. *Advances in Experimental Medicine and Biology*.

[3] Guo Q., Goldenberg J. Z., Humphrey C., El Dib R., Johnston B. C. (2019). Probiotics for the prevention of pediatric antibiotic-associated diarrhea. *Cochrane Database of Systematic Reviews*.

[4] Kelly C. R., Fischer M., Allegretti J. R. (2021). ACG clinical guidelines: prevention, diagnosis, and treatment of clostridioides difficile infections. *American Journal of Gastroenterology*.

[5] Goldenberg J. Z., Yap C., Lytvyn L. (2017). Probiotics for the prevention of Clostridium difficile-associated diarrhea in adults and children. *Cochrane Database of Systematic Reviews*.

[6] Chen S. M., Mao J., Chen Z. R. (2018). Effect of probiotics combined with water-soluble dietary fiber on prevention and treatment of antibiotic-associated diarrhea in elderly. *Tianjin pharmaceutical*.

[7] Liu H., Xu X. L., Zhang R. (2017). Advances in laboratory testing for *Clostridium difficile* infection. *Chinese Journal of Infection Control*.

[8] Nyankovsk Y. S., Nyankovska S., Yatsula M. S. (2020). Features of the use of probiotics for antibiotic-associated diarrhea in children. *Child`S Health*.

[9] Ma X. Y., Yu N., Zhang J. (2017). Analysis of susceptibility factors for antibiotic associated diarrhea in elderly patients. *Chongqing med*.

[10] Ma H., Zhang L., Zhang Y., Yu L., Yingli H., Litao G. (2019). Combined administration of an-tibiotics increases the incidence of antibiotic-associated diarrheain critically ill patients. *Infection and Drug Resistance*.

[11] Feng A. M., Yang H. X. (2019). Effects of different probiotics on intestinal microflora and proinflammatory factors in neonates with antibiotic-associated diarrhea pneumonia. *Chinese Journal of Microecology*.

[12] Liu D., Jiang X. Y., Zhou L. S., Hong S. J., Zhang X. M. D. (2016). Effects of probiotics on intestinal mucosa barrier in patients with colorectal cancer after operation: meta-analysis of randomized controlled trials. *Medicine*.

[13] Liu Y. P., Shi H., Li H. (2018). Effects of probiotics on bacterial community structure and mucosal barrier function in patients with viral diarrhea. *Chinese Journal of Preventive Medicine*.

[14] Giuliano S., Guastalegname M., Russo A. (2017). Candida endo-carditis: systematic literature review from 1997 to 2014 and a-nalysis of 29 cases from the Italian Study of Endocarditis. *Expert Rev Anti Infect Ther*.

[15] Mei C. H., Lu K., Sun L. L. (2018). Effects of probiotics on intestinal microbiota distribution after helicobacter pylori eradication. *Chinese Journal of Microecology*.

[16] Wieërs G., Verbelen V., Van Den Driessche M. (2021). Do probiotics during in-hospital antibiotic treatment prevent colonization of gut microbiota with multi-drug-resistant bacteria A randomized placebo-controlled trial comparing Saccharomyces to a mixture of lactobacillus, bifidobacterium, and Saccharomyces. *Frontiers in Public Health*.

